The article "Pro-Poor Hydraulic Governmentality: Sustainable Water Management and Local Livelihoods in Mekong Delta" was published in 2023. Journal: J Environ Public Health.

# Pro-Poor Hydraulic Governmentality: Sustainable Water Management and Local Livelihoods in Mekong Delta

**DOI:** 10.1155/2023/6739550

**Published:** 2023-02-14

**Authors:** Jinsheng Jason Zhu, Zhiyong Liu

**Affiliations:** ^1^Belt and Road International School, Guilin Tourism University, Guilin 541006, Guangxi, China; ^2^International Hospitality Management, Taylor's University, Subang Jaya 50250, Malaysia

## Abstract

This article considers and adds empirical nuances to the recent conceptualization of pro-poor water management. Using the concept of pro-poor hydraulic governmentality along the Vietnam-Cambodia border of Thường Phước commune, we argue that water management is linked to local rural livelihoods in a complex and dynamic pro-poor mechanism. While certain policies organize local populations according to cost-effectiveness ignoring local customs, the practicalities of dealing with such constraints are much more ambivalent. This article demonstrates the structural pro-poor complexity among sand excavation, riverbank landslides, water management, local livelihoods, and populace resettlement. The government's resettlement plans and the perceptions of residents of these plans are intertwined with a wider political, economic, social, and cultural significance in the context of strong institutional power in Vietnam. Limitations and future research agenda are also indicated in the discussion and conclusion section.

## 1. Introduction

The Mekong Delta is located in the southern part of the Indochina Peninsula [1], straddling Cambodia and Vietnam, with its apex around Phnom Penh, Cambodia. The area has the highest population density and highest per capita income in Vietnam [2]. The Mekong Delta has a tropical monsoon climate with high temperatures throughout the year, clear dry and rainy seasons, and fertile soil suitable for agricultural production [3]. The terrain in this area, low and flat, has dense water networks contributing to fertile farmland. Endowed with these features, the Mekong Delta has a long history of rice cultivation and is the region with the highest rice yield in Asia. Consequently, the Mekong Delta has developed into a densely populated area with about 50 million people. The main cities in the Mekong Delta are Hồ Chí Minh City (Vietnam), Can Tho (Vietnam), and Phnom Penh (Cambodia).

As the rice basket of Vietnam, the Mekong Delta has been constantly facing a couple of constraints brought about by the impact of climate change [4]. For example, sand mining activities increase the risk of riverbank landslides near the Mekong River basin [5–8]. The riverbed mining has long contributed to the increase of an average of 1.3 meter depth of the riverbed, which led to the augmentation of over 400 locations of riverbank erosion and 66% of the foreshore eroding in the Mekong Delta, of which the occurrence is still increasing [9]. This article setting off from the impending phenomenal challenges tries to apply a transdisciplinary approach to examine the hydraulic governmentality theory and investigate the intrinsic networks among the impact of landslides, sand extraction, the governmental resettlement scheme, and the dam-building upstream of the Mekong River. It is hoped that this transdisciplinary research would facilitate a comprehensive understanding of the pro-poor structural complexity of landslides, environmental migration, agricultural adaptability, water management, and farming sustainability in the Mekong Delta. It is also intended to investigate whether or not adaptive knowledge generation and government resettlement policies have a mutually reinforcing impact. The present article concludes that the resilience of citizens' livelihoods and the generation of adaptive knowledge must be included in the effectiveness of a water management system.

The article "Pro-Poor Hydraulic Governmentality: Sustainable Water Management and Local Livelihoods in Mekong Delta" was published in 2023. Journal: J Environ Public Health.

## 2. The Mekong Delta and Hydraulic Governmentality

Considering its geological uniqueness and geographical disposition in the Mekong Delta, we investigate this region using a transdisciplinary approach and propose that water management is related to local livelihoods through complex and dynamic mechanisms, forming a systematic geopolitical network. Water management in the Vietnamese Mekong Delta has been recently described in terms of hydraulic governmentality [10], building on a conceptual fusion of Wittfogel's theory of the hydraulic state [11, 12] and Evers' theory of the formation of strategic groups in Southeast Asia [13]. To build a transdisciplinary development model of pro-poor prevention and mitigation measures, this article will look at the building, restructuring, and renewing of the hydraulic state in one representative commune in Vietnam. Based on this line of thinking, we provide a broader interpretation of hydraulic governmentality [14]. This enables us to extend its usefulness, transcend disciplinary divides, and get beyond some of the despotic and technocratic undertones of the concept's historical contexts. We argue that hydraulic management is not only related to but also encompasses and implies population management which includes quite monolithic top-down approaches as much as micropolitics of conducts.

Existing threats to landslides in addition to the Mekong River have long been characterized by global warming, changing extreme climates (typhoons and heavy storms) and sea level rise, the proliferation of hydroelectric dams in upper regions, excessive excavation of sand in the stream, improper construction of dams in flood plains, as well as other anthropic impacts [15]. This article is structured as follows: Initially, the issues of the Mekong Delta are introduced, followed by a discussion of water management. Second, the article provides a summary of the literature assessment concerning the theoretical examination of hydraulic governmentality and hydraulic state building. The article then describes the rural region of Thường Phước commune, Vietnam, as the study location and presents the research questions. Following more investigations and methodical discussions, we come to the conclusion section.

The article "Pro-Poor Hydraulic Governmentality: Sustainable Water Management and Local Livelihoods in Mekong Delta" was published in 2023. Journal: J Environ Public Health.

## 3. Case Study: Landslides in the Thường Phước Commune, Vietnam

### 3.1. Research Methodology and Research Questions

The research methodologies are mainly on a qualitative approach [16–18], including participatory and nonparticipatory observation, formal and informal focal group interviews, and timeline mapping, as well as theoretical discussion of government documentaries [19]. The initial research question started by brainstorming some core fundamentals surrounding the households affected by landslides, including the reasons for landslides, the implementation of disaster management policies, the resilience of local livelihoods, and the policies related to resettlement plans. We initially schemed a tentative framework, putting the landslide issue as our core focus, taking the political, economic, ecological, historical, and social/cultural approaches into the study, which determined our research methodology and guided us through our empirical data collection, reflexive analysis, and drafting tentative reports. This research project was carried out with two runs of interviews and fieldworks, each of which lasted for 7 days of grounded fieldwork runs from 2019 to 2020 in Thường Phước commune, Vietnam. Systematic interviews were conducted in the Lower Mekong Basin to evaluate the types of materials extracted, the techniques used, the volumes extracted, the trends recorded in recent years, and the expected changes in the geography of river sand extraction. A transect on the walk to the farmland, the river dyke, the channel, and the households in the commune allowed us to meet with more than 38 farmers in 15 families affected by the landslide. We also organized five semiofficial interview meetings with multilevel government officials, including the chief of the commune and deputy chief, the committee member and governors of the Tong Phuc No. 1 commune, the governor of the Department of Agriculture and Rural of Cầu Hồng Ngự, the Department of Resources and Environment in Đồng Tháp province, as well as some higher-level governors in the province, who also facilitated our in situ research fieldwork with official approval documents (for academic purpose) documents. Each of the focal group meetings consisted of 20–15 participants. Unfortunately, we could not interview the sand mining company representatives since sand mining activities are pretty sensitive issues, especially in this area. Based on our preresearch data collections, we brainstormed some frequently asked questions and drafted out the guidelines and those challenges we might face in the field, Thường Phước commune. Thus, we reached a consensus on tentative research questions as follows:

1. What are the reasons that cause the landslides and how do these landslides affect the livelihood of locals in Thường Phước commune's local community?
2. How does the resettlement plan scheme out as countermeasures of resilience and what is the progress of resettlement implementation?
3. To what extent do the multifacet counter-disaster measurement policies instill into the local communities' self-salvation and livelihood resilience to combat the increasing impact of climate change in the Mekong Delta?

The article "Pro-Poor Hydraulic Governmentality: Sustainable Water Management and Local Livelihoods in Mekong Delta" was published in 2023. Journal: J Environ Public Health.

Bearing these research questions in mind, we started collecting some elementary data from the research field, the Thường Phước commune. By investigating the landslide-affected cases in Thường Phước commune, we propose the key argument that landslides as natural disasters are related closely to the efficiency of the water management system, agricultural adaptation, and rehabilitation, as well as the government's intervention policies, especially under the context of Vietnam, a government with a strong structural power hierarchy.

### 3.2. Socioeconomic Background and People's Livelihoods

The research site was Thường Phước commune, Hồng Ngự district, Đồng Tháp province, Vietnam (Figure 1). The commune was established in 2004 by the provincial government as a community affected by landslides. Đồng Tháp province is 145 kilometers southwest of Hồ Chí Minh City. Our research site is located in the Cầu Hồng Ngự district of Đồng Tháp province, covering an area of 209.73 km and sharing an 18-kilometers border with Cambodia. Located in the Mekong Delta region of the Lower Mekong River, this place is featured with a relatively flat terrain, a tropical monsoon climate with equatorial characteristics, and a dense river and canal network. In particular, the Tien River divides the territorial space into two parts: the northern part of the low-lying area of Đồng Tháp and the southern part is sandwiched between the Tien and Hau rivers. Accordingly, Đồng Tháp has many favourable conditions for socioeconomic development, especially water and soil resources. This province, however, also faces many difficulties and challenges from the natural environment, which can be proven in their cultural relics of worshipping their ancestors' heroic efforts to prevent or against natural disasters, such as cemetery building, or in their sincere following of Christianity or Buddhism to pray for God's blessing. The research was conducted in the Thường Phước commune which shares a borderline with Cambodia, covers 547 hectares of land, and has a population over 3000 residents. This commune shares a common tropical climate with 2 seasons, a typical Mekong delta climate. The months from May to November are considered the rainy season and December to April the dry season. The main priorities of economic development and the main products in the commune are fisheries, agriculture (rice and cash crops, such as tuber, cassava, sesame, and chilly plantations), cross-border trade, production of commercial goods, and ecotourism. The Tien River, one of the downstream sections of the Mekong River, flows from Cambodia to Vietnam, among which is the Thường Phước commune, where its waterways take the shape of nine dragons as they make their way to the sea.

The article "Pro-Poor Hydraulic Governmentality: Sustainable Water Management and Local Livelihoods in Mekong Delta" was published in 2023. Journal: J Environ Public Health.

The Mekong Delta, which is dominated by rice plantations and production [20], provides Vietnam with more than half of its rice production, most of its fishing outcomes, and 75% of its fruit plantations [21]. It plays an important role in both domestic food supply and commodity exports in Vietnam. As many as 17 million people are living in the Mekong Delta, which accounts for more than 26% of Vietnam's overall population [22, 23]. For a long time, people have lived on both sides of the river and the canal that the river extends. The management of water resources is a significant topic that cannot be divorced from the social and economic growth of the Mekong Delta as well as the fundamental safety of the people's living conditions.

## 4. Research Analysis on the Impact of Landslides on Local Livelihoods

### 4.1. Landslides in the Mekong Delta

In the Mekong Delta region, residents constantly faced with the impact of various forms of natural disasters; the most distinctive natural disasters were riverbank landslides and fluctuating flash floods. For instance, landslides are devastating natural forces constantly threatening the livelihood of human beings in the Mekong Delta [15, 24, 25]. Monsoon season and dry seasons' rotation have altered the Mekong River swell with kilometer-wide torrents on the riverbanks, scouring soils and sands and houses away. Residents affected have been rehabilitated from riverside areas to faraway resettlement areas. A riverside fishery, livelihood, and the constant splashing water flows and waves over the riverbanks were prone to be easily affected by natural disasters like floods and landslides, causing damage to the destruction of planted crops, sweeping away the infrastructure and displacement of local residences. High and intensive annual rainfalls in the microclimatic features of the Mekong Delta have diversified implications for the downstream Mekong Delta agricultural ecological system. Storms, following the floods, constantly splash over the riverbanks beside the Mekong River. Due to a variety of reasons, this region is easily prone to the reoccurrence of riverbank landslides and flash floods. Devastating landslides threaten local livelihoods, destroying cash crops and rice and leaving infrastructure damaged and local residences displaced. Thus, there is an urgent demand to stabilize the riversides, regulate the annual water inflation, rehabilitate the local livelihoods, and increase the land nutrition balance and production capacity. Throughout the process of household mobilization, a series of land-use schemes have been introduced to tackle the local economic deficiency and develop a sustainable development model. It is then a crucial urge to empower the local people with a sustainable agricultural ecological plantation system or introduce an alternative farming model to facilitate the farming security of the local people. This article thus starts with a discussion of landslides' impacts on the localities. The Tien riverbank has long been affected by floods, dry season erosion, and faced with severe landslide issues. Landslides alongside the Mekong riverbank, however, have long been a devastating and threatening reason for the house collapses in the Thường Phước commune. In recent years, five major landslides have occurred, respectively, in the years 2000, 2008, 2011, 2014, and in August 2018, threatening the livelihoods of the residents. This does not mean that the other years are not affected. The continued impacts of landslides have drastically affected the security of local villagers' households, leaving the local houses with collapsing grounds and falling walls and bricks. Most of the Thường Phước commune villagers' houses were built beside the road along the riverbank. The road itself serves as a barrage to resist the Mekong river's water overflowing into the farmland. Half of the commune houses are adversely threatened or adversely damaged by landslide issues, which are more than 25 kilometers along the riverbank on the east side of the Mekong river. Many landslides occur about 1–3 meters below the household soil, threatening more than 300 hectares of farmland as well as the resident's houses. In this Thường Phước commune, more than a hundred households are located in the endangered area.

The article "Pro-Poor Hydraulic Governmentality: Sustainable Water Management and Local Livelihoods in Mekong Delta" was published in 2023. Journal: J Environ Public Health.

There are extensive concerns about hydropower dams in the upper stream causing the decreasing volume of mud and sands flowing from upstream of the Mekong River. Kummu and Varis [26] proposed a theoretical analysis of the hydropower dams' impact on the total suspended solids decrease due to the sediment concentration in the reservoir [26]. As Nguyen Huu Nhan and Nguyen Ba Cao have pointed out, if

*All the proposed mainstream hydropower dams in the Lower Mekong Basin were built, and then the Vietnamese Mekong Delta with its ecosystems and about 18 million people face critical issues of sustainability* [9].

The construction of hydropower dams is also deemed as a threatening factor in modifying the annual flood height, shortening flood duration, and postponing the flood timing, as well as the sediments. The uncertainty of the water flow and the reduction of sediment projections are also key factors for the adaptation to climate changes in the Mekong Delta [27]. The increasingly extreme weather and the rising of sea levels due to the global warming system are also posing challenges to the downstream of the Mekong River. Illegal sand excavation in Đồng Tháp province has had a dramatic impact on the landslide issues, partially due to Vietnam's economic development and booming construction demands in recent years. The booming demand for construction materials in Vietnam prompted a gradual increase in the volume of construction sand and gravel, which triggered a series of consequences, one of the most distinctive phenomena is illegal sand mining. Increasing mining and excavation of sand has become the fundamental cause of increasing riverbank erosion, which consequently leads to severe landslide threats to the residences beside the Mekong River, especially on our research site, the Thường Phước commune. Some parts of the houses entirely disappeared due to sand and soil subsidence, leaving the remaining houses heavily leveraged. Illegal sand mining has caused serious land subsidence from the riverbanks to the riverbeds, and subsequently, led to irreversible devastation to the local communities.

*My coffee shop used to stand 25 meters away from the river. However, now, as you can see, the river is right underneath my coffee shop. Probably it will disappear within 5 years*. (The interview was conducted in the year 2019 while the authors were doing field visits to the research sites. A coffee shop owner in Vietnam's Thường Phước commune shared his worries about the receding riverbank across the Mekong River in the interview.)

The article "Pro-Poor Hydraulic Governmentality: Sustainable Water Management and Local Livelihoods in Mekong Delta" was published in 2023. Journal: J Environ Public Health.

This comment shows that sand mining is becoming one of the most influential reasons for the constant impacts of landslides. The local people are mainly living beside the Mekong River, which is richly endowed with abundant fishes, including species such as Blackfish and *Catlocarpio siamensis*. The Lower Mekong Delta accounts for as high as 80% of the locals' annual animal protein intake, which is worth around 3 billion USD/year for the productive wetland fishery industry [28]. The fishery industry in Vietnam accounts for 32% of the annual fish catch in the Mekong River, reaching an annual volume of 840,000 tons [29]. Thus, regardless of the challenge of the landslides, the fishermen were continuously building houses beside the easily affected riverbanks. In the dry season, the water erosion effects also threaten the riverbanks. Riverbank erosion in Đồng Tháp province mainly occurs in the rainy season, especially in the flood years. However, in recent years, erosion has occurred more in the dry season (where disputes occur between the upper and tidal currents). In general, river erosion in Đồng Tháp province is increasing both in size and degree of erosion and is related to complicated development issues. Due to the lack of prevention measurements of water erosion techniques, there is no soil and water conservation besides the Mekong riverbank. The study of morpho dynamics of the eroding riverbanks in the Mekong River delta implies that the deltaic sand erosion could be happening even more severely during the dry season when the river level is lower than usual. The soil sediment erosion effect seems again to be largely related to both the upper stream (China, Thailand, and Lao PDR) water flow and the lower (western part of Vietnam) regions [30]. Another reason for dry season water/soil erosion was a lack of budget and the government's relocation to build dykes beside the riverbanks.

*Compared with relocating residents to the resettlement area, building stone and concrete dykes on the riverbanks is more costly. In consideration of the cost-benefit results, we prefer to move people, rather than sparing our budget by building dykes.* (Interviewed the *representing* administrative of the township of Vietnam's Thường Phước commune in 2019, who expressed the resettlement plan initiated by the Vietnam local government of Đồng Tháp province, Vietnam).

Thus, even though the local communities are still facing houses losing solid ground in their backyards, they have to use reality and withstand the threats.

### 4.2. Analysis of Sand Extraction in the Mekong River

The extraction of river sand and gravel has increased in developed countries since at least the middle of the twentieth century, in particular for the construction of concrete and embankments. In the last 30 years, this phenomenon has expanded greatly in developing countries, especially the fast-growing Vietnam in the lower Mekong Delta. The negative impacts of river resource extraction have been extensively examined in the Lower Mekong Basin and its impacts over tributary basins are hotspots of biodiversity. The reasons most often cited for the decline of the delta riverbanks are the trapping of sediments in the reservoirs of the upper river. The extraction of sand and gravel in the Mekong riverbed and its tributaries also affected the river waves. The results reveal that the annual volume of sand and gravel extracted, despite obvious underestimation, exceeds the volume of sand and gravel transported by the river. The results also underline the considerable importance of this factor in the geomorphological and ecological changes recorded in the different sections of the Mekong and its delta. The impact of sand excavation in the past was far more than imagination. According to Vietnam news, both legal and illegal sand mining ships have been booming in the Mekong River since the year 2000, digging deep into the riverbed to excavate sands for increasing construction demands. Roaring dredging boats use rackety pumps to dig into the riverbed and drag out an enormous amount of the indispensable commodity in concrete-sand for construction [31]. Most of the sand ships constantly operate in areas as close as 50 meters to the riverbanks. In 2016 alone, for instance, the Vietnamese police caught nearly 3,000 people dredging without permits or in protected areas around the country [31]. In the Thuong Phuoc commune, being aware of the severance of negative impact of sand mining on household safety, the local communities organized an outbreak of protests against the illegal sand excavation ships, which indirectly led to a batch of government officials in jail, for bribe-taking from the illegal sand excavation companies before 2013. To tackle the existing landslide problems, systematic countermeasures as this should be taken into consideration.

The article "Pro-Poor Hydraulic Governmentality: Sustainable Water Management and Local Livelihoods in Mekong Delta" was published in 2023. Journal: J Environ Public Health.

## 5. Key Perceptions and Resolutions for Locals to Cope with Landslide Issues in the Lower Mekong Delta

Facing these challenges, this article proposes the application of the theory of hydraulic governmentality as countermeasures for a better water management system.

### 5.1. Dilemmatic Understanding of Sand Excavation and Solution

In this special research site, we found that both the government and the local communities are now agreeable to sand excavations since the new regulations set a 300-meter offshore borderline to the riverbank, much more than the previous 50 meters before 2013. After the new regulation's implementation, there is a consensus in this specific commune that the riverbed in the middle of the Tien River will become deeper, which will lead to the water flow becoming less influential and reducing the splashing power to the riverbanks. One of the key informants from a local authority, who is also a hydraulic expert, mentioned that

*Sand excavation in the middle of the riverbed made it deeper from the previous 5-6 meters to more than 10 meters, which facilitates larger cargo ships to go bypass, to some extent, it helps us with international business connecting the upper and downstream Mekong river countries as far as Thailand and Lao PDR.* (The interview was done in the year 2019 in the focus group discussion with one of the key informants from a local authority, who is also a hydraulic expert in the province).

Another local tradesman expressed his concern about the big waves that the cargo ships create, saying that the

*Container ships' engine motors create big waves, splashing more stronger on the riverbanks. To us, this is one of the other threatening reasons for landslides b*esides the riverbank. (In the year 2019, an interview was conducted with a local businessman who expressed his concerns over the large waves that are caused by cargo ships passing by in the Mekong River).

According to our observations and the results of the face-to-face interview, sand mining is a societal issue that is extremely severe and a substantial contributor to environmental degradation over time. Even if the likelihood of landslide concerns is reduced, the sand dome that is forming on the other side is sending tremendous waves to the riverbanks. Sand from the island is taken away by each river wave that smashes on the dune and wipes it away, leading small business owners along the river to experience distress, as well as the possible threats of environmental degradation and landslides.

### 5.2. Complex Perceptions over the Resettlement Plan and Residence Mobilization

To deal with the existing problems for the landslide-affected houses, over the past 20 years, the Vietnam government has planned and carried out a household resettlement project. Between 2012 and 2013, up to 292 households had to be resettled in the resettlement area. Back in 2008, 36 households were removed from the riverbank. As early as 2002, 151 households were forced to be resettled. However, there are still 192 households that remain threatened in the landslide-threatening area. During the time we conducted the research, we found that there were perplexed perceptions over the resettlement plans between the local community and the government, sometimes even contradicting each other.

The article "Pro-Poor Hydraulic Governmentality: Sustainable Water Management and Local Livelihoods in Mekong Delta" was published in 2023. Journal: J Environ Public Health.

### 5.3. The Government's Role in the Resettlement Scheme

The local government simplified the solution for landslide-victimized households. In the context of Vietnam, a society with a strong hierarchy, the government exerts its hegemonic power in the governance of political, social, and cultural issues, especially in current research backdrops, emphasizing the economic reform since 1985. The structural mechanism of the government requires the government to be more responsive to engaging with landslide-affected households, restricting over-cultivation to the farmlands, implementing empowerment training programs for farmers, and carrying out more efficient resettlement policies. During the meeting with the provincial governors, they mentioned that the Vietnam government proposed funding support with a VND house-building loan ranging from one to twelve million to the resettled families to build houses in the resettlement area. The loan can be postponed by paying it back after 5 years. The repayment would be prolonged to more than 10 years, which to some extent eased the financial burden of the resettled household. This district suffered from a devastating flood in 2000 when the river level rose to a historically heigh level of more than 6 meters, washing lots of houses away. Accordingly, the resettlement plan was initially proposed in 2001 and started to be implemented in 2002, when more than 150 households were successfully resettled. The following years witnessed a consecutive impact of floods and the resettlement plan continues. An important premise of household resettlement is the construction of basic service facilities, such as electricity, water supply, and transporting roads, as well as community rehabilitation facilities such as schools, hospitals, and healthcare organizations. The necessary living facilities, such as schools, hospitals, and the construction of the daily consuming market were the leg behind the needs of the resettled communities so far. Similar to the solutions proposed by Young [32], institutional dynamic mechanisms should be implemented to accumulate and escalate the adaptation capacity of the local communities under the ever-changing environmental influences condition. Therefore, systematic collaboration among governments, cooperatives, both wealthy and poor households, and construction houses is needed for successful rehabilitation to be implemented. The establishment of proper regulations might take time to negotiate. It is, however, extremely crucial for the governance mechanism to achieve the sustainable development of the whole resettlement plan.

The article "Pro-Poor Hydraulic Governmentality: Sustainable Water Management and Local Livelihoods in Mekong Delta" was published in 2023. Journal: J Environ Public Health.

### 5.4. The Consensus Reached by Environmental Migrants over How to Deal with Landslides

Landslides are complexly relevant to human environmental displacement. In Vietnam, environmental displacement is interwoven with socioeconomic factors, which is consistent with stakeholder disagreements, disputes, and conflicts [33]. Yamamoto [34] examined the multiple drivers of displacement and Vietnamese government policies as counter-measurements [34]. The displaced local communities could be classified as one of the forms of environmental migrants as they are displaced by the forces of natural disasters. Migration of this kind, due to the deterioration of the natural environment on which people depend, are referred to as the environmental migration [35]. Ecological migration is an environmental movement induced by ecological environment deterioration such as desertification and soil erosion [36]. Causes contributing to environmental migration include natural disasters, ecological degradation, environmental pollution, and other environmental factors [36]. Following this, environmental disaster migrations are migrations induced by natural disasters such as floods, droughts, mudslides, and landslides. Local residents of our study site are compelled to abandon their houses and relocate to the new resettlement location. Thus, their sense of participating in the resettlement plan is ambiguous and divided. In our research field visits, we found that there are complex reasons for the landslide households to move or not move to the resettlement area. Both the pros and cons are taken into consideration.

### 5.5. The Pros to the Resettlement Scheme for the Landslide-Affected Residents

Such people are displaced due to the construction of dams or the destruction of households by natural disasters, which might be exacerbated by inadequate or poorly planned infrastructure. In the household visit to the resettled area, an interviewee pointed out that

*We were initially reluctant to move here because the resettlement is 10 kilometres from my house beside the river. Even though the landslide endangers the house, we have our farmland beside our house. It is pretty inconvenient for us to commute for cultivation and agricultural activities. In addition, my previous home is still in fairly good condition, and my daughter attends the local community school. Therefore, I am much preferring to keep my daughter continue staying in our cottage back on the riverside, staying with her grandparents*. (During the household visit in the resettled region, an interviewee expressed his thoughts on his forced relocation from his original residence to the resettled household. The interview was conducted during the second field visit undertaken in the year 2020).

The article "Pro-Poor Hydraulic Governmentality: Sustainable Water Management and Local Livelihoods in Mekong Delta" was published in 2023. Journal: J Environ Public Health.

Social and cultural values are also needed to be considered in the perceptions of the reluctance of joining the resettlement plan. Ancestor worship in Vietnam is an extremely strong tradition that has lasted for years. Thus, the graveyards of passed away ancestors are buried right beside the houses or farmland. The offspring's values are largely determined by their care for the ancestor's graveyard. Some of the local residents are largely related or determined by their livelihoods and personal diseases or by the influence of the buried ancestors' cemetery. One of the interviewees whom we met in the resettled area mentioned that

*We moved to this new settlement zone in 2018. We were unable to move from the landslide areas because my father strongly refused and debuted the government's proposal of resettlement. It was until he passed away that our family was able to start the moving process. That was why we moved here so late. Yet my mother is still staying in my old house, caring for my past away father's cemetery. Once she left the old house and lived here in the resettlement zone, she started to get severe sickness. I believe it was because my past-away father does not happy to see her leaving the old house*. (In 2018, one of the respondents in the resettled region stated that they were forced to relocate to the new settlement zone. Previously, they were unable to leave the landslide zones since my father flatly rejected and denounced the government's relocation plan.)

This sounds like a superstitious belief, yet the local values of land nostalgia and a sense of belonging are greatly attached to the farmland they cultivate, as well as the houses they lived in for years, especially those houses of their ancestors. The existence of ancestor worship has extensive popularity among the residents. Thus, it is also a hard choice for them to move. The sense of belonging still needs to be taken into consideration in the resettlement process.

### 5.6. The Cons to the Resettlement Scheme for the Landslide-Affected Residents

However, some of the families we interviewed were pretty happy with the resettlement plan. For example, one middle-aged woman expressed her satisfaction with the resettlement community,

*I was pretty happy with the resettlement. Since my washed-away house in the landslide disaster did not register in the household registration system, we lost everything in the floods. With the support of the government, we took a loan from the government and rebuilt our new house in the resettlement area. What makes me happier was that by now I could officially register my household in the registration system*. (The interview was conducted in 2020 when the authors visited the research sites in the fieldwork. The respondent, a middle-aged lady, was satisfied with the resettlement community).

The article "Pro-Poor Hydraulic Governmentality: Sustainable Water Management and Local Livelihoods in Mekong Delta" was published in 2023. Journal: J Environ Public Health.

Similar to China's Hukou system, Vietnam's household registration identifies each person as a rural or urban resident with a permanent or temporary registry [37, 38]. It is essential for managing population mobility and determining eligibility for state-provided services and social support [39]. A nonregistered resident to a registered resident joining the resettlement arena was an enticing option for these families, allowing them to send their children to nearby schools and get access to the social ware fare system with educational opportunities, healthcare, and employment generation.

### 5.7. The Complex Perceptions over the Landslide-Related Mekong Delta Annual Floods

Local stakeholders' perceptions of the ecoagricultural system are far more diversified and complex in the Mekong Delta in Vietnam [40]. Changing the functionality of land use leads to soil nutrition degradation in the downstream Mekong River. Due to the desire to maximize rice productivity, the local government was constantly investing to build solid embankments and waterways to exert the maximum usage of the land, prevent flooding, and cultivate 3 crops a year. The plantation scheme also has a strong link with flood-affected rehabilitation to increase the capacity to combat the landslides' negative impact and increase the adaptability to regional climate change. Engaging in diversified cash crops could also help residents to manage increasingly extreme climates. It is a strong necessity to ensure a sustainable usage of farming land and agricultural biodiversity in this area. Despite the dominance of rice plantations throughout the region, the Mekong Delta has long been introducing a vibrant bio-diversified planting system to ensure land nutrition safety by introducing supplementary cash crops like sesame, tuber cassava, tangerine, and vegetable crops, which serve as an alternative biodiversity related to agricultural safety. These implementations also increased the adaptability of the local residents to the increasing climate changes. In our field visit to Thường Phước commune, a villager from the farmer's association mentioned that

*Our commune's farmlands are a bit higher than the other communes, that is the reason our local authority invested to build a higher dyke to prevent annual flooding. We are glad to see these embankments. However, we gradually realized that continuous 3-season rice plantations would lead to land nutrition degradation, which will lead to lower productivity*. (Interviewed in 2019).

The article "Pro-Poor Hydraulic Governmentality: Sustainable Water Management and Local Livelihoods in Mekong Delta" was published in 2023. Journal: J Environ Public Health.

Regardless of the prospect of lower productivity, the local villagers are also more prone to plant 3 crops a year.

*By planting 3 crops a year, we could gain 60 million VND per hectare, without the third planting season, we could only gain approximately 40 million*. (Interviewed in 2019).

The local rice plantation knowledge also makes them realize that it is more feasible to plant 2 seasons of rice and one season of cash crops, such as sweet potato, tuber, cassava, and sesame, for better preservation and recovery of land nutrition. There are plans to take advantage of floods (such as dredging canals and digging water canals) for deacidification, washing saline, alum, and cleaning fields. Changing crop structure, especially in the autumn and winter (season 3), from sole rice production in areas where there are permanent dykes and other areas that could cultivate short-term crops to avoid floods. Currently, the rice crop structure is shown in Table 1. It should be noted that the autumn-winter crop was actively sown and conducted an early harvest before the floods came.

Furthermore, an expert from Cần Thơ University in Vietnam, Mr. Le Anh Tuan, has mentioned in one interview, “*the farmers can breed fish in flooding season in Đồng Tháp province*” [42], which proposes a traditional solution to the stress of annual flooding of the Mekong Delta. In our interview with the governor in charge of the administration of Thuong Phuoc Commune People's Committee, the interviewee stated the World Bank project was a planned project for the vision of sustainable development in the Mekong Delta. The World Bank project provides a development perspective on the resilience of local communities to better adapt to natural disasters. Another project, supported by the International Climate Initiative (IKI) of the Federal Ministry for the Environment, Nature Conservation, Building, and Nuclear Safety (BMUB) in Germany, was established from January 2017 to December 2020. The Mekong WET program aimed at enhancing the resilience capacity of wetlands in the downstream Mekong Delta by harnessing the benefits from four countries: Cambodia, Thailand, Lao PDR, and Vietnam.

### 5.8. Self-Salvation and Empowerment of Local Livelihoods to Combat Landslides

The lower Mekong Delta has long been impacted by floods and landslides for years, which have caused severe losses in human beings, households, transportation facilities, and the agricultural sector. The vulnerability of human beings under constantly increasing extreme weather is often neglected. With its strong institutional and structural hierarchical power in Vietnam, the government is constantly providing overall counter-measurements within the scope of the existing landslide risk management framework. However, while we conducted face-to-face interviews both with middle- and higher-ranking officials in Đồng Tháp province, as well as victim individuals affected by landslides, self-salvation as a solution was frequently raised in the discussion. It is similar to what Luu et al. [43] have proposed that, while the flood risk management activities in Vietnam are implemented according to the hierarchical structure of the political system and the responsibilities of various paramount government agencies, there is an urgent need for experts, researchers, and scientists participating in the decision-making steering committee, most importantly, there is even more urgent need for greater public participation at local levels [43]. The locals bear a much more profound knowledge to understand their life situations. Thus, the empowerment strategy for flood mitigation would be a necessity to put in the overall landslide rehabilitation scheme. Empowerment programs would be needed to implement landslide-impacted household resilience.

The article "Pro-Poor Hydraulic Governmentality: Sustainable Water Management and Local Livelihoods in Mekong Delta" was published in 2023. Journal: J Environ Public Health.

*Climate change adaptation capacity could not rely solely on outer forces. It is crucial for the farmers and residents, whose households were affected, to enhance their capacity for climate change adaptation. The ultimate solution should be generated from their strength. It is themselves that they should rely upon much* (interviewed in 2020).

Another villager who we interviewed also expressed his reliance attitude:

*Floods came every year; landslides are also a constant threat to our houses. If we only lay at home and waited for government assistance, we could not increase our life quality. That is for sure* (Interviewed in 2020).

Vogel and Meyer [44] proposed a similar concept on how to increase the adaptation capabilities to secure food production security under climate extremes in agricultural sectors [44]. The cause of the hazards is the combined impact of natural factors (mainly) and socioeconomic activities that are not rational in the basin and locality, contributing to the increase of disasters (in terms of extent and damage). Thus, even though Đồng Tháp province is facing all kinds of disasters such as floods, riverbank erosion, droughts, and intrusions, which are also causing damage to people and property, hindering the sustainable socioeconomic development of the province, it is much more necessary to facilitate and increase the residents' self-rehabilitation capacity and enhance their wellbeing using their capabilities.

To realize this vision, the stakeholder's involvement in the empowerment process has been extensively studied in academics, which is also examined in Timothy's (2004) empowerment and stakeholder debate. He analysed that the power struggles have been and will continue to be part and parcel of everyday life in most parts of the world. Unfortunately, as they continue, the most disadvantaged groups, such as ethnic and racial minorities, women, and the poor, remain the most powerless (cf. [45]: 212). In doing so, integrating the local farmer's adaptive knowledge has become crucial for a better water management system and adaptive policy implementation in Vietnam [46]. Empowerment over marginalized groups regardless of an ethnic minority, a biased gender, or the communities and individuals that are affected and excluded by the benefits of social and urban development brought about by or affected by natural calamities like river-flood-caused landslides, would be of crucial importance. However, cultural and political obstacles and equal beneficiary disposition under the highly structured Vietnam context still exist in crucial at all levels of the scale decision-making process on resettlement planning and implementation. Economic deficiencies and government budgets restrain a portion of the stakeholders from benefiting equally from the profit gained from the respected margin. The voice of equilibrating power of a marginalized group of people is barely enough, and a true implementation to exercise real practical empowerment to the stakeholders in the resettlement sector and landslide resilience has become an impending urgency in modern Vietnam society. Moreover, psychological empowerment over the related parties could also initiate positive feedback in terms of relation construction among the government, the local community, and the residents. Stakeholder empowerment would cast its influence over livelihood settlement, legislative governance, agricultural commodity production and consumption, as well as overall water management effectiveness in the resilience schema.

The article "Pro-Poor Hydraulic Governmentality: Sustainable Water Management and Local Livelihoods in Mekong Delta" was published in 2023. Journal: J Environ Public Health.

## 6. Discussion and Conclusions: Pro-Poor Hydraulic Governmentality

Governmentality, as is shown by its literate meaning, connotates those well-organized practices (mentality, rationality, and technique) through the governed subjects (populaces, people, and individuals) [47, 48]. In the case of societies that highly rely on water resources, water governmentality could be one of the leading guidelines for reaching a balanced social structure as well as building stable hydrological territory [49, 50].

Coming back to the Thường Phước commune in this article, in light of the hydraulic governmentality, we could raise this argument: well-structured water resources management is crucially essential to local livelihoods in a complex and dynamic mechanism. Thinking through the concept of hydraulic governmentality, several key summaries can be found in the abovementioned discussion:

1. Landslide-sand mining nexus: one might conclude that sand mining may cause riverbank landslides, while others might not think this way. A deeper pursuit of the resettlement plan might be safer for the citizens in riverbed eroded banks.
2. Hydraulic dam-building: The contested understanding is manifested within the process of conceptualizing, decision-making, designing, constructing, developing, and governing those mega-hydraulic infrastructures in the Mekong region.
3. Governance rationality: To govern a hydrosociety requires a gradual and emerging process towards rational, cobenefit governance by applying rational sociotechnical, adaptive, and flexible strategies.
4. Water management—at times this may be shown in very twisted ways, such as by not developing the waterfront but instead resettling people. Villagers are differently affected by landslides and populace resettlement.
5. Self-salvation: in a society under hydraulic bureaucracy governance, the flows of water are equal to the flows of power. It is the mission of a highly structured state water governmentality to enhance and strengthen the countermeasures for self-process and inner-generated livelihood improvement via proper empowerment endeavours.

The discussions above have shown that water management is one of the crucial issues for the resilience of landslide-affected communities. Building dynamic land use and integrated hydrological water control infrastructures are deemed effective ways of combating the threatening landslide issues. That is the reason Vietnam aimed at building a hydrological state, both integrating the land-use and hydrological regime [51]. By applying a transdisciplinary approach to understanding the situations about livelihood resilience, we could determine that applying different theories in the research is a convenient method to identify the prime problems and figure out the action plan. Flooding is helping with local farming, or is it devastating forces on the livelihood of the locals? We need to apply the transdisciplinary approach, putting environmental governance as the core focus. Referred to as diversified stakeholders, academic knowledge, hydraulic experts, institutional capacity, government policy-makers, and local people's empirical experience all work together to figure out the prime concern of the landslide-affected resident's livelihood and resilience. To proactively prevent and mitigate damages caused by natural disasters in the locality, Đồng Tháp province needs to implement solutions guided by both the strongly structured government and the people themselves. As each solution has its advantages and disadvantages, it is necessary to coordinate solutions in the implementation process to ensure the highest efficiency. In the immediate future, the province should prioritize the construction of flood-prone residential clusters and routes, the construction of embankments, and relocation of people in the areas that occur and where there is a risk of high river erosion to limit human damage and the loss of property. Furthermore, certain remedial measurements and solutions could also decrease, but not thoroughly eliminate, the negative influences of the proposed middle- and lower-stream dams in the Mekong Basin in Vietnam. By exerting people's active role in combating the negative impacts of natural disasters, we could cross the boundary of disciplinary boundaries, generalize a certain common conceptualization of the landslide as a research object, and structure a new framework of theory and discovery. To answer the perception of a sustainable water management system, we could conceptualize the environmental governance issues with the following framework, taking into consideration the three mechanisms, namely, the government's role, the ecological impacts, and the human activities intervening as the following chart (see Figure 2) shows.

The article "Pro-Poor Hydraulic Governmentality: Sustainable Water Management and Local Livelihoods in Mekong Delta" was published in 2023. Journal: J Environ Public Health.

The framework urges a free flow of data sharing, transparent decision processing, and inclusive transnational environment governance in the Mekong Delta, water management, addressing issues of the global environment, e.g., resilience to climate change), natural resources (e.g., wetlands ecosystems), local environmental quality, local competence, local awareness, living with floods, recognizing the benefits of floods, as well as zoning and relocation (e.g., striking a balance between the risk of living in endangered flood plains and sociocultural stress management) [53]. There is an urgent demand to apply a transdisciplinary research approach to determine proper initiatives for the resilience of the landslide-affected communities, increasing their adaptability to the increasing impacts of climate change as well as the political, cultural, and socioecological impacts, and ultimately reaching a balanced and sustainable water management system.

## Figures and Tables

**Figure 1:** Map of Đồng Tháp province. Đồng Tháp is one of 12 provinces in the Mekong Delta. It is about 165 km from Hồ Chí Minh city and shares the same border with Cambodia in the north, Vĩnh Long, and Cần Thơ in the south. The pink section is the district of Cầu Hồng Ngự, Vietnam, where the Tien river (one part of the mainstream Mekong River) flows from Cambodia into Vietnam (Source: https://mekongsmiletour.com/what-to-do-in-dong-thap/).

The article "Pro-Poor Hydraulic Governmentality: Sustainable Water Management and Local Livelihoods in Mekong Delta" was published in 2023. Journal: J Environ Public Health.

**Figure 2:** The pro-poor water management model in the environmental governance approach, which integrates the ecological and human activity mechanisms and the impacts forces value systems. It produces a systematic framework to integrate three categories of driving forces, taking the Mekong Delta's pro-poor water management as the core concern. (The figure is inspired by and adapted from the transdisciplinary theory of researchers Bruno Messerli and Paul Messerli [52]).

**Table 1:** Rice crop structure (3 crops) in Đồng Tháp Province ( Source: [41]). Information was also collected from the interview with representatives from the farmer's association in Thường Phước commune, Đồng Tháp province, in 2019.

Plantation service	Time of plantation	Harvest time	Note
Winter-spring	September 5–1 November	February-March	Should only be planted in areas with solid embankments, if not converted to growing cash crops or short-term industrial plants, and vegetables.
Summer-autumn	February-March	May-June	
Autumn	In June	In September	

## Data Availability

The data used to support the findings of this study are included within the article.

## Additional Points

*Highlights*. (1) The complexity of social structure, environmental migration, agricultural adaptation, and water management contribute to the sustainability of livelihood in the Mekong Delta. (2) Studies on adaptive knowledge production and government resettlement policy have a mutual reinforcement effect. (3) Resilience to the livelihood of residents and the production of adaptive knowledge must be integrated into the efficiency of a water management system.
